This article has been retracted.

# Two Different Transplant Preconditioning Regimens Combined with Irradiation and Chemotherapy in the Treatment of Childhood Leukemia: Systematic Review and Meta-Analysis

**DOI:** 10.1155/2022/2825712

**Published:** 2022-03-18

**Authors:** Xiangwen Wang, Dan Mu, Anyang Geng, Anqi Zhao, Yiyuan Song

**Affiliations:** Inner Mongolia People's Hospital Pediatric Hematology, Hohhot, China

## Abstract

**Objective:**

To observe the therapeutic effect and the incidence of adverse reactions of total body irradiation plus cyclophosphamide (TBI/CY) and busulfan plus cyclophosphamide (BU/CY) in the treatment of pediatric hematopoietic stem cell transplantation.

**Methods:**

By searching the Cochrane Library, PubMed, Web of Knowledge, Embase, Chinese Biomedical Literature Database (CBM), and screening randomized controlled trials (RCTs), quality evaluation and data extraction were performed for the included literature, and meta-analysis was performed for RCTs included at using Review Manager 5.2 software.

**Results:**

A total of 10160 patients were enrolled in 15 RCTs, including 5211 patients in the TBI/CY group and 4949 patients in the BU/CY group. Meta-analysis showed that there was a statistical difference in transplant failure rate (OR = 1.56, 95% CI (1.23, 1.97), *P* = 0.0002, *I*^2^ = 56%, *Z* = 3.69), transplant mortality (OR = 1.45, 95% CI (1.24, 1.68), *P* < 0.00001, *I*^2^ = 76%, *Z* = 4.80), transplantation long-term disease-free survival rate (OR = 1.52, 95% CI (1.09, 2.12), *P* = 0.01, *I*^2^ = 0%, *Z* = 2.50), and transplantation adverse reactions (OR = 1.28, 95% CI (1.08, 1.52), *P* = 0.004, *I*^2^ = 0%, *Z* = 2.85).

**Conclusion:**

Meta-analysis showed that TBI/CY combined pretreatment regimen was more effective than BU/CY regimen alone in the treatment of pediatric hematologic transplantation, with a lower incidence of adverse reactions and significant long-term survival efficacy.

## 1. Introduction

Acute leukemia (AL) is a heterogeneous malignant clonal disease of hematopoietic stem cells, with a high recurrence rate and mortality rate [1]. Leukemia is mainly because of hematopoietic stem cells during differentiation and infiltrating the tissues and organs of the human body. Then, it caused different degrees of fever, anemia, and bleeding symptoms [2–5]. Leukemia has a high incidence of pediatric malignant tumors, mostly presented as acute leukemia. Nowadays, with the gradual improvement of clinical hematopoietic stem cell technology and hematopoietic stem cell source, the success rate of transplantation is significantly improved, making more children with leukemia have the desire for long-term survival [6].

Pediatric leukemia is a high incidence of malignant tumor in China [7]. Currently, although allogeneic hematopoietic stem cell transplantation (allo-HSCT) can serve as an effective treatment for AL, patients of leukemia still face various complications after transplantation, including graft-versus-host disease(GVHD), venoocclusive disease (VOD), thrombotic microvascular disease (TMA), and fungal infection that have caused adverse effects on the survival and prognosis of AL patients after transplantation. The main measures for the clinical treatment of the disease include chemical therapy, targeted therapy, and hematopoietic stem cell transplantation. For children with refractory and recurrent leukemia, conventional chemotherapy is short [8]. Nowadays, with the continuous in-depth research of the clinical characteristics of hematopoietic stem cells and transplantation immune technology and the continuous promotion of new anti-infectious drugs and immunosuppressors, bone marrow transplantation has been gradually developed and improved, and now, it has become one of the main means for the treatment of hematological diseases. Acute leukemia is characterized by abnormal proliferation of leukemia cells, abnormal primitive cells, and naive cells in the bone marrow, which can be widely infiltrated into the extramedullary organs, and is clinically manifested by different degrees of anemia, bleeding, infection, and other symptoms. Allogeneic HSCT is currently the main treatment for hematological malignancies, but the recurrence rate after acute leukemia transplantation is still not significantly reduced. Studies at home and abroad show that if small residual disease can be detected before transplantation, the recurrence rate of patients is significantly increased after transplantation, but there are few survival studies on myeloablative HSCT [9].

Allogeneic hematopoietic stem cell transplantation (Allo-HSCT) is the preferred method for treating AML in middle and high-risk patients, and the quality of the pretreatment regimen directly affects the prognosis of patients. Traditional busulfan combined with cyclophosphamide (BU/CY) and total body irradiation combined with cyclophosphamide (TBI/CY) protocol. Guolo et al. [10] showed that overall and leukemia-free survival had significant advantages for patients undergoing pretreatment with systemic radiotherapy in remission, but large meta-analysis showed similar survival for the two regimens. Therefore, for relapsed/refractory acute myeloid leukemia resistant to multiple chemotherapy drugs, a systemic radiotherapy myelination-based regimen might be needed. Whether conditioning regimen, it has an advantage that has not been explicitly recommended.

Therefore, in this study, relevant randomized controlled trials in recent years were systematically searched, and meta-analysis was used to evaluate the efficacy and safety of two different transplant preconditioning regiments combined with radiotherapy and chemotherapy in the treatment of childhood leukemia, providing reliable evidence for clinical treatment.

## 2. Materials and Methods

### 2.1. Search Strategy

In this study, Cochrane Library, PubMed, Web of Science, Embase, and CBM were searched and other databases and related websites search. Subject words such as “Transplant,” “Total body irradiation,” “Busulfan,” “Childhood leukemia,” “Cyclophosphamide,” and related drug trade names were retrieved as subject words and free words, respectively. In order to avoid bias caused by language limitations, this study searched both Chinese and English literature. In order to avoid missing relevant studies, relevant references listed in the article and conference abstracts found in the search were traced (Figure 1).

### 2.2. Data Extraction

Data extraction was completed independently by two evaluators. First, read the title of the literature, read the abstract of the literature related to the content of this study, and further read the full text of the literature if it is a randomized controlled trial. The studies that met the inclusion and exclusion criteria were classified and evaluated, and the data were extracted. If there is any disagreement between the two reviewers in the selection of literature, the problem will be solved through discussion within the group. The authors of studies for which detailed data were not available were contacted by e-mail or by reviewing the literature referencing the candidate study. The inclusion criterion is childhood diagnosed with leukemia, aged 1–14 years. The exclusion criterion is patients treated with irradiation and chemotherapy before.

### 2.3. Literature Quality Assessment

2 reviewers used the Jadad rating scale to independently evaluate 15, mainly to evaluate the randomized controlled experimental design of the included literature, including generation of random sequence (“yes” = 2, “unclear” = 1,“ no” = 0); random hiding (“yes” = 2, “unclear” = 1,“ no” = 0); blind (“yes” = 2, “unclear” = 1,“ no” = 0); and exit (“yes” = 1, “no” = 0). A score of 1–3 is considered low quality, while a score of 4–7 is considered high quality. Data extraction of information mainly includes the author information, country, Jadad score, types and patient's age and gender, study drug dosage, number of cycles, effective treatment before and after treatment, and adverse reaction condition, after data extraction, two commentators' data comparison, discuss the inconsistencies, and supplement the missing information as much as possible.

### 2.4. Bias Analysis

Heterogeneity between studies was assessed using *I*^2^ statistics, 25%, 50%, and 75% representing low, medium, and high heterogeneity, respectively; *I*^2^ < 50% and *P* > 0.1 between studies using fixed effect models and *I*^2^ > 50% and *P* < 0.1 from chi-square analysis showed study heterogeneity. Meta-analysis was done by random effects models and searched for possible heterogeneity by subgroup analysis source. The sensitivity analysis removed the included literature one by one to see whether the pooled effect values were stable and reliable (Figures 2 and 3).

### 2.5. Statistical Analysis

Consolidated effect size analysis of indicators of concern for this system evaluation was analyzed using STATA 12.0 software. For measurement data, the weighted mean difference (WMD) is the same; the standard mean difference (SMD) and its 95% CI are the effect amount. Relative hazard (relative risk, RR) and its 95% CI were used as the effect size, and *P* < 0.05 was used as the statistical difference. Intertest heterogeneity was performed using a 2-test, *P* > 0.1, and *I*^2^ <50%. If there is no heterogeneity, the fixed effect model is used for data pooled analysis, and the random effect model for pooled analysis and subgroup analysis was to detect the reasons for possible clinical heterogeneity and statistical heterogeneity. Publication bias was detected by the rank correlation test (Begg method) and the linear regression method (Egger method). Finally, the sensitivity analysis was conducted by the elimination method to test the stability of the results level. For the meta-analysis, there must be treatment effects and their standard deviation.

## 3. Result

### 3.1. Basic Characteristics of Literature

A total of 802 documents were initially retrieved, and duplicates were removed by software with 692 remaining. After reading of the topic, abstract, and full text, 15 literature [11–25] were obtained, and a total of 10160 patients were included in the meta-analysis, including 5211 in the TBI/CY group and 4949 in the BU/CY group. Final included general features of the 15 literature are given in Table 1.

### 3.2. Transplant Failure Rate

Among the 15 RCTs literature included in transplant failure rate, the heterogeneity test was carried out, and it was found that the heterogeneity of the selected studies was small, so meta-analysis with fixed models could be performed. The results of meta-analysis showed that the rhombus plot and vertical line not intersected in the forest map of transplant failure rate for 4 included literature, so there was a statistical difference in the comparison of transplant failure rate between the BU/CY group and the TBI/CY group (OR = 1.56, 95% CI (1.23, 1.97), *P* = 0.0002, *I*^2^ = 56%, *Z* = 3.69) (Figure 4).

### 3.3. Transplant Mortality

Among the 15 RCTs literature included in transplant mortality, the heterogeneity test was carried out, and it was found that the heterogeneity of the selected studies was small, so meta-analysis with fixed models could be performed. The results of meta-analysis showed that the rhombus plot and vertical line not intersected in the forest map of transplant mortality for 4 included literature, so there was a statistical difference in the comparison of transplant mortality between the BU/CY group and the TBI/CY group (OR = 1.45, 95% CI (1.24, 1.68), *P* < 0.00001, *I*^2^ = 76%, *Z* = 4.80) (Figure 5).

### 3.4. Transplantation Long-Term Disease-Free Survival Rate

Among the 15 RCTs literature included in the transplantation long-term disease-free survival rate, the heterogeneity test was carried out, and it was found that heterogeneity of the selected studies was small, so meta-analysis with fixed models could be performed. The results of meta-analysis showed that the rhombus plot and vertical line not intersected in the forest map of transplantation long-term disease-free survival rate for 4 included literature, so there was a statistical difference in the comparison of transplantation long-term disease-free survival rate between the BU/CY group and the TBI/CY group (OR = 1.52, 95% CI (1.09, 2.12), *P* = 0.01, *I*^2^ = 0%, *Z* = 2.50) (Figure 6).

### 3.5. Incidence of Transplantation Adverse Reactions

Among the 15 RCTs literature included in incidence of transplantation adverse reactions, the heterogeneity test was carried out, and it was found that the heterogeneity of the selected studies was small, so meta-analysis with fixed models could be performed. The results of meta-analysis showed that the rhombus plot and vertical line not intersected in the forest map of incidence of transplantation adverse reactions for 4 included literature, so there was a statistical difference in the comparison of incidence of transplantation adverse reactions between the BU/CY group and the TBI/CY group (OR = 1.28, 95% CI (1.08, 1.52), *P* = 0.004, *I*^2^ = 0%, *Z* = 2.85) (Figure 7).

## 4. Discussion

Pretreatment protocol of allo-HSCT for AML, retrospective analysis, and meta-analysis had no clear answer as to whether TBI treatments are superior to BU treatment. It has been shown that oral BU in TBI-MAC patients reduced relapse rate and disease-free survival is high; while, patients treated with intravenous BU, with improved survival due to reduced side effects of BU, obtained similar results to that of TBI-MAC. Analysis from the International Blood and Bone Marrow Transplantation Research Center showed that for AML patients in remission, disease-free and overall survival in the BU group outperformed the TBI group, with similar relapse rates and low nonrelapse mortality [26]. No large sample size has been reported in treating similar results in AML patients with relapse/refractory. The statistical results from this study showed that relapse was the main cause of death in the two groups of relapsed/refractory AML patients. In addition to applying new drugs and new technologies to reduce the pretransplant tumor load, the improved pretreatment protocol can also reduce the nonrelapse mortality and improve survival. In recent years, it has been reported that pretreatment with TBI combined with BU or mafalan has reduced nonrelapse mortality and improved disease-free survival in patients. At the same time, the residual leukemia was detected regularly after transplantation, and the early withdrawal of immunosuppressant and immunotherapy also improved according to the patient's disease status and patient prognosis [27].

Hematopoietic stem cell transplantation can cure childhood leukemia, aplastic anemia, hemoglobin disease, and congenital immune deficiency [28]. The pretreatment regiments for pediatric transplantation include total body irradiation (TBI) and chemotherapy alone [29–32]. The most classical pretreatment regiments are TBI/CY and BU/CY. Preconditioning is one of the important factors affecting the curative effect of hematopoietic stem cell transplantation [33]. The BU/CY-based pretreatment protocols are two of which are considered classical pretreatment options for HSCT [34]. However, there is little literature on the impact of different pretreatment protocols on pediatric HSCT [35]. The results show that children in hematopoietic stem cell transplantation, TBI/CY and BU/CY two pretreatment methods, implant failure rate, no significant difference between the BU/CY group-related increased mortality after transplantation, might be more prone to this group of patients after transplantation of complications such as complicated with hepatic vein occlusion disease, hemorrhagic cystitis, and lead to the early death of increase after transplantation. The long-term disease-free survival rate in the TBI/CY group was significantly better than that in the BU/CY group [36–39].

This study has some limitations: the number of RCTs included and the number of cases is small, which may have a certain publication bias; the number of included literature was small, and no subgroup analysis was performed to compare the efficacy; this study only evaluated the efficacy at the end of treatment, but did not evaluate the maintenance of the medium and long-term efficacies.

## 5. Conclusion

The available evidence tentatively demonstrates the safety and efficacy of BU/CY in pediatric HSCT [40], and TBI/CY combined pretreatment regimen was more effective than BU/CY regimen alone in the treatment of pediatric hematologic transplantation, with a lower incidence of adverse reactions and significant long-term survival efficacy.

## Figures and Tables

**Figure 1:** Flowchart of the literature screening.

**Figure 2:** Literature quality evaluation chart. (a) Risk of bias graph. (b) Risk of bias summary.

**Figure 3:** (a)–(d) Funnel plot of literature publication bias.

**Figure 4:** Meta-analysis of transplant failure rate between two groups.

**Figure 5:** Meta-analysis of transplant mortality between two groups.

**Figure 6:** Meta-analysis of transplantation long-term disease-free survival rate between two groups.

**Figure 7:** Meta-analysis of incidence of transplantation adverse reactions between two groups.

**Table 1:** Basic clinical features of 15 literature included in our study.

Study	Age	Gender (male) (%)	Hospitalization days	BU/CY group (*N*)	TBI/CY group (*N*)	NOS score	Research type
Speziali et al. [11]	6.71 ± 2.2	44.25	17.8 ± 1.1	26/146	16/146	8	RCT
Uberti et al. [12]	6.65 ± 3.4	59.12	12.2 ± 1.3	240/1593	200/1593	7	RCT
Bernard et al. [13]	6.12 ± 4.5	45.72	12.4 ± 3.9	174/240	66/130	7	RCT
Salhotra et al. [14]	7.15 ± 1.5	44.12	12.9 ± 4.9	47/167	34/167	7	RCT
Kalaycio et al. [15]	6.85 ± 2.4	51.89	9.8 ± 3.4	19/86	14/86	8	RCT
Copelan et al. [16]	6.36 ± 3.2	63.45	11.2 ± 5.1	311/1230	197/1230	7	RCT
Bernard et al. [17]	9.62 ± 12.2	78.10	10.9 ± 2.1	16/42	14/46	9	RCT
Guilcher et al. [18]	6.61 ± 3.0	48.75	19.9 ± 1.4	21/78	17/78	9	RCT
Scott et al. [19]	7.25 ± 1.51	59.23	13.4 ± 4.1	43/128	40/128	7	RCT
De Berranger et al. [20]	6.22 ± 1.21	56.22	17.8 ± 1.5	56/226	41/142	8	RCT
Bredeson et al. [21]	11.35 ± 2.12	53.16	16.1 ± 5.9	121/458	102/458	8	RCT
Cahu et al. [22]	9.25 ± 1.01	66.34	17.5 ± 1.6	125/601	112/601	8	RCT
Dahlke et al. [23]	8.51 ± 2.61	48.34	15.0 ± 5.6	23/76	16/76	7	RCT
Bonini et al. [24]	12.34 ± 3.51	53.12	12.4 ± 1.7	12/26	9/26	9	RCT
Granados et al. [25]	9.25 ± 4.21	67.22	11.1 ± 1.2	45/114	11/42	9	RCT

## Data Availability

The data used to support the findings of this study are available from the corresponding author upon request.

## References

[1] Cunningham I. (2021). Post-transplant leukemia relapse in organs: biology. and behavior in 585 reports. *Critical Reviews in Oncology*.

[2] Rautenberg C., Germing U., Haas R., Kobbe G., Schroeder T. (2019). Relapse of acute myeloid leukemia after allogeneic stem cell transplantation: prevention, detection, and treatment. *International Journal of Molecular Sciences*.

[3] Dholaria B., Savani B. N., Hamilton B. K. (2021). Hematopoietic cell transplantation in the treatment of newly diagnosed adult acute myeloid leukemia: an evidence-based review from the American society of transplantation and cellular therapy. *Transplantation and Cellular Therapy*.

[4] Yeo K. K., Kayser K., Margol A. S. (2019). Clinical and neuropsychological outcome of pediatric non-midline central nervous system germinoma treated with chemotherapy and reduced dose/volume irradiation: the Children’s Hospital Los Angeles experience. *Pediatric Blood & Cancer*.

[5] Lulla P. D., Naik S., Vasileiou S. (2021). Clinical effects of administering leukemia-specific donor T cells to patients with AML/MDS after allogeneic transplant. *Blood*.

[6] Scobioala S., Eich H. T. (2020). Risk stratification of pulmonary toxicities in the combination of whole lung irradiation and high-dose chemotherapy for Ewing sarcoma patients with lung metastases: a review. *Strahlentherapie und Onkologie*.

[7] Guillaume T., Malard F., Magro L. (2019). Prospective phase II study of prophylactic low-dose azacitidine and donor lymphocyte infusions following allogeneic hematopoietic stem cell transplantation for high-risk acute myeloid leukemia and myelodysplastic syndrome. *Bone Marrow Transplantation*.

[8] Li C., Ni W., Wang X. (2019). A phase I/II radiation dose escalation trial using simultaneous integrated boost technique with elective nodal irradiation and concurrent chemotherapy for unresectable esophageal Cancer. *Radiation Oncology*.

[9] Olson A. L., Saliba R. M., Oran B. (2021). Cytogenetics and blast count determine transplant outcomes in patients with active acute myeloid leukemia. *Acta Haematologica*.

[10] Guolo F., Di Grazia C., Minetto P. (2021). Pre‐transplant minimal residual disease assessment and transplant‐related factors predict the outcome of acute myeloid leukemia patients undergoing allogeneic stem cell transplantation. *European Journal of Haematology*.

[11] Speziali C., Daly A., Abuhaleeqa M. (2019). Fludarabine, busulfan, and low-dose TBI conditioning versus cyclophosphamide and TBI in allogeneic hematopoietic cell transplantation for adult acute lymphoblastic leukemia. *Leukemia and Lymphoma*.

[12] Uberti J. P., Agovi M.-A., Tarima S. (2011). Comparative analysis of BU and CY versus CY and TBI in full intensity unrelated marrow donor transplantation for AML, CML and myelodysplasia. *Bone Marrow Transplantation*.

[13] Bernard F., Auquier P., Herrmann I. (2014). Health status of childhood leukemia survivors who received hematopoietic cell transplantation after BU or TBI: an LEA study. *Bone Marrow Transplantation*.

[14] Salhotra A., Hui S., Yang D. (2020). Long-term outcomes of patients with acute myelogenous leukemia treated with myeloablative fractionated total body irradiation TBI-based conditioning with a tacrolimus- and sirolimus-based graft-versus-host disease prophylaxis regimen: 6-year follow-up from a single center. *Biology of Blood and Marrow Transplantation*.

[15] Kalaycio M., Bolwell B., Rybicki L. (2011). BU- vs TBI-based conditioning for adult patients with ALL. *Bone Marrow Transplantation*.

[16] Copelan E. A., Hamilton B. K., Avalos B. (2013). Better leukemia-free and overall survival in AML in first remission following cyclophosphamide in combination with busulfan compared with TBI. *Blood*.

[17] Bernard F., Bordigoni P., Simeoni M.-C. (2009). Height growth during adolescence and final height after haematopoietic SCT for childhood acute leukaemia: the impact of a conditioning regimen with BU or TBI. *Bone Marrow Transplantation*.

[18] Guilcher G. M. T., Moorjani R., Truong T. H., Lewis V. A. (2015). Myeloablative BU, fludarabine, antithymocyte globulin and low-dose TBI in the treatment of juvenile myelomonocytic leukaemia with allogeneic haematopoietic cell transplantation. *Bone Marrow Transplantation*.

[19] Scott B., Deeg H. J., Storer B. (2004). Targeted busulfan and cyclophosphamide as compared to busulfan and TBI as preparative regimens for transplantation in patients with advanced MDS or transformation to AML. *Leukemia and Lymphoma*.

[20] De Berranger E., Cousien A., Petit A. (2014). Impact on long-term OS of conditioning regimen in allogeneic BMT for children with AML in first CR: TBI+CY versus BU+CY: a report from the Société Française de Greffe de Moelle et de Thérapie Cellulaire. *Bone Marrow Transplantation*.

[21] Bredeson C., LeRademacher J., Kato K. (2013). Prospective cohort study comparing intravenous busulfan to total body irradiation in hematopoietic cell transplantation. *Blood*.

[22] Cahu X., Labopin M., Labopin M. (2016). Impact of conditioning with TBI in adult patients with T-cell ALL who receive a myeloablative allogeneic stem cell transplantation: a report from the acute leukemia working party of EBMT. *Bone Marrow Transplantation*.

[23] Dahlke J., Kröger N., Zabelina T. (2006). Comparable results in patients with acute lymphoblastic leukemia after related and unrelated stem cell transplantation. *Bone Marrow Transplantation*.

[24] Bonini A., Bandini G., Rosti G. (1998). Big BU/CY is associated with a favorable long-term outcome in patients allotransplanted for chronic myelogenous leukemia in chronic phase. *Bone Marrow Transplantation*.

[25] Granados E., de La Cámara R., Madero L. (2000). Hematopoietic cell transplantation in acute lymphoblastic leukemia: better long term event-free survival with conditioning regimens containing total body irradiation. *Haematologica*.

[26] Marino L., Lancellotta V., Franco P. (2021). Loco-regional adjuvant radiation therapy in breast cancer patients with positive axillary lymph-nodes at diagnosis (CN2) undergoing preoperative chemotherapy and with complete pathological lymph-nodes response. Development of GRADE (Grades of recommendation, assessment, Development and Evaluation) recommendation by the Italian Association of radiation therapy and Clinical Oncology (AIRO). *The Breast*.

[27] Lehrnbecher T., Averbuch D., Castagnola E. (2021). 8th European Conference on Infections in Leukaemia. 8th European Conference on Infections in Leukaemia: 2020 guidelines for the use of antibiotics in paediatric patients with cancer or post-haematopoietic cell transplantation. *The Lancet Oncology,*.

[28] Al-Shaibani E., Cyriac S., Chen S. (2021). Comparison of the prognostic ability of the HCT-CI, the modified EBMT, and the EBMT-ADT pre-transplant risk scores for acute leukemia. *Clinical Lymphoma, Myeloma & Leukemia*.

[29] Groll A. H., Pana D., Lanternier F. (2021). 8th European Conference on Infections in Leukaemia: 2020 guidelines for the diagnosis, prevention, and treatment of invasive fungal diseases in paediatric patients with cancer or post-haematopoietic cell transplantation. *The Lancet Oncology*.

[30] Burgos-Burgos J., Vega V., Macias-Verde D. (2021). Hypofractionated whole breast irradiation after IORT treatment is safe in patients receiving adjuvant chemotherapy. *Clinical and Translational Oncology*.

[31] Lu Y., Hua J., Yan F. (2021). Combined radiotherapy and chemotherapy versus radiotherapy alone in elderly patients with nasopharyngeal carcinoma. *Medicine*.

[32] Yegin Z. A., Can F., Gökçen S. (2020). The impact of pre-transplant cell-free DNA levels on leukemia relapse and transplant-related complications in allogeneic hematopoietic stem cell transplant recipients. *Balkan Medical Journal*.

[33] Ho V. T., Martin A. S., Pérez W. S. (2020). Prior gemtuzumab ozogamicin exposure in adults with acute myeloid leukemia does not increase hepatic veno-occlusive disease risk after allogeneic hematopoietic cell transplantation: a center for international Blood and marrow transplant research analysis. *Biology of Blood and Marrow Transplantation*.

[34] El Fakih R., Savani B., Mohty M., Aljurf M. (2020). Hematopoietic cell transplant consideration for philadelphia chromosome-like acute lymphoblastic leukemia patients. *Biology of Blood and Marrow Transplantation*.

[35] Elsharawi R., Antonucci E., Sukari A., Cramer J. D. (2021). Quality metrics for head and neck cancer treated with definitive radiotherapy and/or chemotherapy. *Head & Neck*.

[36] Loke J., Buka R., Craddock C. (2021). Allogeneic stem cell transplantation for acute myeloid leukemia: who, when, and how?. *Frontiers in Immunology*.

[37] Salas M. Q., Prem S., Atenafu E. G. (2019). Reduced intensity allogeneic stem cell transplant with anti‐thymocyte globulin and post‐transplant cyclophosphamide in acute myeloid leukemia. *European Journal of Haematology*.

[38] Kongtim P., Parmar S., Milton D. R. (2019). Impact of a novel prognostic model, hematopoietic cell transplant-composite risk (HCT-CR), on allogeneic transplant outcomes in patients with acute myeloid leukemia and myelodysplastic syndrome. *Bone Marrow Transplantation*.

[39] Morisaki T., Ohguri T., Yahara K. (2021). Salvage Re-irradiation with intensity-modulated radiotherapy, chemotherapy combined with hyperthermia for local recurrence of nasopharyngeal carcinoma after chemoradiotherapy. *Journal of UOEH*.

[40] Muffly L. (2019). Transplant for acute myeloid leukemia in patients aged 70 Years and older: optimism and opportunity. *Biology of Blood and Marrow Transplantation*.

